# Overexpression of Peanut Diacylglycerol Acyltransferase 2 in *Escherichia coli*

This article has been retracted.

**DOI:** 10.1371/journal.pone.0061363

**Published:** 2013-04-11

**Authors:** Zhenying Peng, Lan Li, Lianqun Yang, Bin Zhang, Gao Chen, Yuping Bi

**Affiliations:** 1 High-Tech Research Center, Shandong Academy of Agricultural Science, Jinan, China; 2 Shandong Provincial Key Laboratory of Crop Genetic Improvement, Ecology and Physiology, Jinan, China; 3 College of Life Science, Shandong Normal University, Jinan, China; University of Nottingham, United Kingdom

## Abstract

Diacylglycerol acyltransferase (DGAT) is the rate-limiting enzyme in triacylglycerol biosynthesis in eukaryotic organisms. Triacylglycerols are important energy-storage oils in plants such as peanuts, soybeans and rape. In this study, *Arachis hypogaea* type 2 *DGAT* (*AhDGAT2*) genes were cloned from the peanut cultivar ‘Luhua 14’ using a homologous gene sequence method and rapid amplification of cDNA ends. To understand the role of AhDGAT2 in triacylglycerol biosynthesis, two AhDGAT2 nucleotide sequences that differed by three amino acids were expressed as glutathione S-transferase (GST) fusion proteins in *Escherichia coli* Rosetta (DE3). Following IPTG induction, the isozymes (AhDGAT2a and AhDGAT2b) were expressed as 64.5 kDa GST fusion proteins. Both AhDGAT2a and AhDGAT2b occurred in the host cell cytoplasm and inclusion bodies, with larger amounts in the inclusion bodies. Overexpression of AhDGATs depressed the host cell growth rates relative to non-transformed cells, but cells harboring empty-vector, AhDGAT2a–GST, or AhDGAT2b–GST exhibited no obvious growth rate differences. Interestingly, induction of AhDGAT2a–GST and AhDGAT2b–GST proteins increased the sizes of the host cells by 2.4–2.5 times that of the controls (post-IPTG induction). The total fatty acid (FA) levels of the AhDGAT2a–GST and AhDGAT2a–GST transformants, as well as levels of C12:0, C14:0, C16:0, C16:1, C18:1n9c and C18:3n3 FAs, increased markedly, whereas C15:0 and C21:0 levels were lower than in non-transformed cells or those containing empty-vectors. In addition, the levels of some FAs differed between the two transformant strains, indicating that the two isozymes might have different functions in peanuts. This is the first time that a full-length recombinant peanut DGAT2 has been produced in a bacterial expression system and the first analysis of its effects on the content and composition of fatty acids in *E. coli*. Our results indicate that AhDGAT2 is a strong candidate gene for efficient FA production in *E. coli.*

## Introduction

Diacylglycerol acyltransferase (DGAT) is the rate-limiting enzyme of the Kennedy pathway for synthesizing triacylglycerols (TAGs) in eukaryotes. DGAT genes have been identified in a wide range of organisms [1]–[4], but TAGs are especially important for energy storage in oil-producing plants, especially peanuts, soybeans and rape. At least four different types of DGAT have been identified in plants. DGAT1 and DGAT2 are transmembrane domain proteins with essential roles in TAG biosynthesis in plants and other eukaryotes [3]. Only one soluble DGAT (DGAT3) has been identified in peanut cotyledons; however, BLAST analyses have identified several potential orthologs in EST collections from *Arabidopsis*, rice, and other plant species [5]. The fourth type, phospholipid:diacylglycerol acyltransferase (PDAT), catalyzes the acyl-CoA-independent formation of TAG in yeast and plants [6]. DGAT1 makes the major contribution to seed oil accumulation [1], [4], [7], whereas DGAT2 and PDAT both affect the specific accumulation of unusual fatty acids (FAs) in seed oil [2], [8]–[11]. These enzymes have unique expression patterns in a variety of plant tissues [7] and may have other roles besides seed oil accumulation, such as FA mobilization [12] and leaf senescence [13]. The process by which such enzymes are regulated in developing seeds and other tissues remains poorly understood.

Much research has focused on DGATs because of their important roles in TAG synthesis. Overexpression of such genes can greatly increase the oil content of transgenic organisms. For example, overexpression of the *Arabidopsis* DGAT1 gene in tobacco and yeast greatly enhanced the TAG content of the transformed lines [14]–[15]. Interestingly, *Ricinus communis* DGAT2 (RcDGAT2) has a strong preference for hydroxyl FAs containing diacylglycerol (DAG) substrates, the levels of which increased from 17% to nearly 30% when RcDGAT2 was expressed in *Arabidopsis* [10]. In *Ricinus* seeds, RcDGAT2 expression was 18-fold higher than in leaves, whereas RcDGAT1 expression differed little between seeds and leaves. Hence, RcDGAT2 probably plays a more important role in castor bean seed TAG biosynthesis than RcDGAT1 [2]. In addition, OeDGAT1 from the olive tree *Olea europaea* is responsible for most TAG deposition in seeds, while OeDGAT2 may be a key mediator of higher oil yields in ripening mesocarps [16].

Recombinant proteins can be used as alternatives to endogenous ones to study their structures and functions or to make high-titer antibodies that recognize them. Because most DGATs are integral membrane proteins, they are difficult to express and purify in heterologous expression systems [17], [18]; thus far, only limited success has been achieved in this area [18]–[20]. Weselake *et al*. expressed the N-terminal 116 amino acid residues of *Brassica napus* (oilseed rape) DGAT1 as a His-tagged protein in *Escherichia coli* [16]. The resulting recombinant BnDGAT1_(1–116)_His_6_ interacted with long chain acyl-CoA and displayed enhanced affinity for erucoyl (22:1cis^Δ13^)-CoA over oleoyl (18:1cis^Δ9^)-CoA [18]. Subsequently, the amino terminal 95 residues of mouse DGAT1 were expressed in *E. coli* with similar results [19]. Encouragingly, full-length DGAT1 expression from the tung tree (*Vernicia fordii*) in *E. coli* has been achieved [20]. In this case, the recombinant protein was mostly targeted to the membranes, and there were insoluble fractions with extensive degradation from the carboxyl end as well as association with other proteins, lipids, and membranes.

*Arachis hypogaea* (peanut, Fabaceae) is one of the most economically-important oil-producing crops, so the fact that peanut DGATs have not been extensively studied is surprising. Saha *et al*. identified a soluble DGAT3 from immature peanut cotyledons and expressed its full length in *E. coli*, where the recombinant protein had high levels of DGAT activity but no wax ester synthase activity [5]; this is the only published report on peanut DGATs thus far. Here, we identified two isozymes of DGAT2 in peanut and expressed both of them as full-length recombinant proteins in *E. coli.* This is the first time that a full-length recombinant DGAT2 protein from peanut has been successfully expressed in *E. coli*, and the first evaluation of its effects on the growth and FA content of the transformed *E. coli* strains studied.

## Materials and Methods

### Cloning of the full-length peanut DGAT2 cDNA

Total RNA (5 µg) from peanut cultivar ‘Luhua 14’ pods obtained 25 days after flowering (DAF) was reverse-transcribed into first-strand cDNAs using a cDNA synthesis kit (Invitrogen, Carlsbad, CA, USA) in a 20 µL reaction volume. Examination of the conserved domains of soybean GmDGAT2 and RcDGAT2 nucleotide sequences enabled us to design a pair of primers (AhD2-S: 5′ TCTTACACCAGCAACAAGGAAA 3′ and AhD2-A: 5′ GACCAAAGCAGAAAACAGGAAC 3′) (Sangon Co., Shanghai, China) that successfully amplified a 197-bp fragment of the gene. The 20 µL PCR mixture contained 1 µL cDNA, 1 µL of each primer (10 µM), 2 µL PCR buffer (10×), 2 µL dNTPs (2.5 mM each), and 1 unit of *Pyrococcus furiosus* (*Pfu*) DNA polymerase (Invitrogen). The reaction was denatured at 94°C for 5 min; followed by 30 cycles of 30 s at 94°C, 30 s at 50°C, and 30 s at 72°C; then 10 min at 72°C. PCR was performed in a PCR Thermal Cycler Dice-TP600 (Takara, Otsu, Japan). The AhDGAT2 fragment was purified using a MinElute™ Gel Extraction Kit (Qiagen, Hilden, Germany), cloned into a pMD18-T vector (Takara), and sequenced.

The full-length AhDGAT2 from ‘Luhua 14’ was cloned using a SMART™ RACE cDNA Amplification Kit (Clontech, Mountain View, CA, USA). Total RNA (1 µg) from the 25-DAF peanut pods was used for cDNA synthesis following the manufacturer's protocol. Rapid amplification of cDNA ends (RACE) primers were based on the sequence of the AhDGAT2 fragment described above as follows: AhD2-3O (5′ TCTTACACCAGCAACAAGGAAA 3′) and AhD2-3I (5′ CCCTCTTGGATAATGGCTACAGTTG 3′), and AhD2-5O (5′ ACTGTAGCCATTATCCAAGAGGG 3′) and AhD2-5I (5′ TTTCTTTGTTGCTGGTGTAA 3′). PCRs were performed according to the manufacturer's protocol. The fragments were sequenced and assembled into a full-length sequence.

Based on the full-length sequence of the AhDGAT2 gene, its full-length open reading frame (ORF) was amplified with gene-specific primers (AhD2-FS: 5′ TCAACAGCCACCGAATCCA 3′ and AhD2-FA: 5′ TAAAACAAGGAAGGGTGCCA 3′). The 20 µL PCR volume comprised 1 µL cDNA, 1 µL of each primer (10 µM), 2 µL PCR buffer (10×), 4 µL dNTPs (2.5 mM each), and 1 unit of *Pfu* DNA polymerase. The reaction was denatured at 94°C for 5 min; followed by 30 cycles of 30 s at 94°C, 30 s at 60°C, and 1 min 20 s at 72°C; then 10 min at 72°C. The full length fragment (AhDGAT2 ORF) was purified from an agarose gel and cloned into a pMD18-T vector for sequencing.

Translations of the full-length ORF sequences were analyzed for structural motifs. Transmembrane helices were predicted using TMHMM (http://www.cbs.dtu.dk/services/TMHMM/), conserved domains were found using the Conserved Domain Database (http://www.ncbi.nlm.nih.gov/Structure/cdd/wrpsb.cgi) at the National Center for Biotechnology Information (NCBI), and putative functional motifs were identified using PROSCAN (http://npsa-pbil.ibcp.fr/cgi-bin/npsa_automat.pl?page=/NPSA/npsa_proscan.html). We also predicted the two- and three-dimensional structures of the genes using phyre2 (http://www.sbg.bio.ic.ac.uk/phyre2/html/page.cgi?id=index).

### Phylogenetic analyses

To better understand the evolutionary origins of the AhDGAT2s, their protein sequences were aligned with those of other DGAT2 genes obtained from NCBI. Homologous sequences in GenBank were identified by a protein BLAST with E-value>6e-149. A multiple sequence alignment using hydrophilic and residue-specific penalties was conducted in DNAMAN 6.0 software (Lynnon Biosoft, Quebec, Canada), which was also used to reconstruct a phylogenetic tree using the observed divergency distance method and default parameters. Two sequences from monocots, *Zea mays* and *Oryza sativa*, were used as outgroups. Statistical support for the tree was gauged using 500 bootstrap replicates.

### Construction of recombinant AhDGAT2a and AhDGAT2b expression vectors and transformations

AhDGAT2a and AhDGAT2b ORFs were amplified using DGAT2a-S2 (5′ CGCGGATCCATGGAAGATCGAGGGAACGT 3′), DGAT2b-S2 (5′ CGCGGATCCATGAAGTCCGAGGGAACGT 3′) and DGAT2-A2 (5′ CCGCTCGAGTCAGACAATTCTCAACTCAAGG 3′) primers, after which the PCR products were restriction digested with *Bam*HI and *Xho*I then ligated into the similarly-digested expression vector pGEX-4T-1 (Biovector Science Lab, Beijing, China) for expression as GST-tagged fusion proteins. The constructs were transformed into the *E. coli* Rosetta (DE3) strain (Transgen, Beijing, China) following the manufacturer's directions.

We evaluated the time course of expression of the fusion proteins by inducing cells transformed with the empty vector or with a GST-tagged fusion protein with 1.0 mM IPTG at 25°C or 37°C. Cells were collected after 0, 2, 4, and 6 h by centrifuging (5,000×g, 10 min), and the pellets were sonicated for 10 min in homogenization buffer (3–4 mL/g wet cells) containing 20 mM Tris-HCl, pH 7.4, 200 mM NaCl, 10 mM β-mercaptoethanol, 1 mM EDTA, 0.5 mM phenylmethylsulfonyl fluoride, and 1∶100–1∶500 dilution of protease inhibitor cocktail (#P8340, Sigma–Aldrich, St. Louis, MO, USA). Cell debris, inclusion bodies, and protein aggregates in the homogenate were removed by two consecutive centrifugations (2,000×g, 10 min, followed by 10,000×g, 10 min). Samples were treated with 0.5 M NaOH and protein concentrations were determined with the Bradford method (Protein Assay Dye Reagent Concentrate, Bio-Rad, Hercules, CA, USA). The supernatant and the pellet were evaluated by SDS-PAGE (10%) and visualized by staining with Coomassie brilliant blue. Furthermore, the expression locations of the recombinant proteins were determined by purifying cytoplasmic and inclusion body fractions using a B-PER GST Fusion Protein Purification Kit (Thermo Scientific, Rockford, IL, USA). Protein expression was verified by a western blot analysis using an anti-GST tag monoclonal antibody (EarthOx, San Francisco, CA, USA).

### Growth and morphology of AhDGAT2a and AhDGAT2b transformed *E. coli* strains

To examine how transformation with DGAT2 affected bacterial growth rate, wild-type (WT) Rosetta (DE3) *E. coli* strains and strains transformed with either empty vector, AhDGAT2a–GST, or AhDGAT2b–GST were cultured in Luria broth (LB) medium at 37°C at an initial density of OD_600_ = 0.05. IPTG (1.0 mM final concentration) was added after 2.0 h for protein induction. OD_600_ measurements were conducted every hour for 8 h using an Evolution 300 spectrophotometer (ThermoFisher Scientific, Waltham, MA, USA). Each treatment was examined in triplicate.

We also evaluated the morphological effects of transformation on these four cell types. At 0, 2, 4, and 6 h after IPTG induction, *E. coli* cells were smeared onto glass slides and heat fixed, after which a drop of crystal-violet Gram staining solution was added. Cells were stained for ∼1 min, washed three times in distilled water, air-dried, then visualized under a light microscope (Zeiss, Jena, Germany) at 1000× magnification under an oil immersion objective. Over 100 cells were observed at each time point in each of three replicates.

### Fatty acid analysis

WT and transformed strains were cultured in liquid LB for 2 h, after which the fusion proteins were induced with 1.0 mM IPTG for 6 h. Isochronous WT cultures and un-induced transformed strains were used as controls. After induction, thalli were collected and freeze-dried for FA analysis. The whole procedure was repeated for a total of two replicates.

Thalli were accurately quantified and soaked in 2.0 mL 2% sulfuric acid in dry methanol for 16 h at room temperature followed by 80 min at 90°C to convert the FAs into FA methyl esters (FAMEs). Supelco™ 37 Component FAME Mix (Sigma–Aldrich, St. Louis, MO, USA) was added as an internal standard. After addition of 2.0 mL of distilled water and 3.0 mL of hexane, the FAMEs were extracted for analysis with a 6890N gas chromatograph (Agilent, Santa Clara, CA, USA). Lipids were measured with a programmed temperature method. An initial column temperature of 140°C was maintained for 5 min, then increased to 240°C at a rate of 4°C/min and held for 10 min. Injection and detector temperatures were 240°C and 260°C, respectively. Two microliters of the sample were injected into the column. FAMEs were identified by comparison of their retention times with those of known standards. The results were analyzed using Chrom Perfect® LSi system software (Fife, Scotland) with the FAME Mix peak area used as the reference.

Fatty acid content was computed as the absolute content (mg/g) using the gas chromatograph area counts for the different FAMEs. The FAME quantity in a sample was used to calculate the oil content using the following equation:





Where M_s_ is the weight of the internal standard added to a sample, A_i_ is the area count of an individual FAME, A_s_ is the area count of the corresponding FAME in the internal standard, and M is the weight of the *E. coli* extract used.

### Statistical analyses

Differences in cell volumes, growth rates, and FA content among the four strains when induced and uninduced were statistically analyzed by one-way analysis of variance (ANOVA) using SPSS 16.0 (IBM, Chicago, IL, USA).

## Results

### Comparison of AhDGAT2a and AhDGAT2b proteins

By employing a homologous gene sequence method with RACE, we identified two isozymes of AhDGAT2 from the peanut cultivar ‘Luhua 14’ and designated them AhDGAT2a and AhDGAT2b (GenBank accession numbers JF897614 and JF897615, respectively). We identified 14 nucleotide differences between them (Figure S1), but the predicted amino acid sequences exhibited only three differences in the N-terminal region (Figure 1). A phylogenetic analysis of the amino acid sequences of the AhDGAT2s and other known DGAT2s (Figure 2) demonstrated that the two AhDGAT2s were closely related to one another and to the DGAT2 from another Fabaceae species (*Medicago truncatula*), to which they exhibited high similarity (91.02%). They were also quite similar to EaDGAT2 from *Euonymus alatus* (Celastraceae; 88.12%).

**Figure 1:** Comparison of the amino acid sequences of AhDGAT2a and AhDGAT2b. The three amino acid differences are shaded in gray. Two black underlined regions (amino acids 40–62 and 67–82) highlight the two predicted transmembrane domains. The red underline shows the conserved LPLAT_MGAT-like domain (amino acids 104–321).

**Figure 2:** Phylogenetic tree showing relationships among the DGAT2 protein sequences from various plant species. The tree was generated using DNAMAN software. Branch lengths indicate evolutionary distance. The GenBank protein ID numbers for the DGAT2s are as follows: MtDGAT2, *Medicago truncatula*, ACJ84867.1; AtDGAT2, *Arabidopsis thaliana*, NP_566952.1; EaDGAT2, *Euonymus alatus*, ADF57328.1; HaDGAT2, *Helianthus annuus*, ABU50328.1; OeDGAT2, *Olea europaea*, ADG22608.1; RcDGAT2, *Ricinus communis*, XP_002528531.1; VfDGAT2, *Vernicia fordii*, ABC94473.1; ZmDGAT2, *Zea mays*, NP_001150174.1; OsDGAT2, *Oryza sativa* Japonica Group, NP_001057530.1. The two peanut DGAT2s are underlined.

The two AhDGAT2s had the same predicted internal structures. Using TMHMM, we identified two potential transmembrane helices, at amino acid positions 40–62 and 67–82 (Figure 1), suggesting that these proteins are located in the membrane system. This program also predicted the presence of a small N-terminal domain and a large C-terminal domain on the cytoplasmic side of the membrane. The Conserved Domain search inferred that both AhDGAT2s possessed an LPLAT_MGAT-like domain at their C-terminus (amino acids 104–321). This domain is a putative acyl-acceptor binding pocket and suggests that AhDGAT2 has acyltransferase activity. PROSCAN identified six putative functional motifs, including N-glycosylation, cAMP- and cGMP-dependent protein kinase phosphorylation, protein kinase C phosphorylation, casein kinase II phosphorylation, N-myristoylation sites, and an amidation site (Table 1). Two putative functional motifs, namely the N-glycosylation (NVTA versus NVTV) and the first N-myristoylation sites, in AhDGAT2a and AhDGAT2b differed because of a mutation at the ninth amino acid position. N-glycosylation is a form of co-translational and post-translational modification. Recently, N-glycosylation of a protein was found to affect its catalytic activity, thermostability, folding, subcellular localization, and secretion, as well as having an impact on pathogen interactions [21]-[24]. N-myristoylation plays a vital role in membrane targeting and signal transduction in plant responses to environmental stress [25], [26]; AhDGAT2a contained four N-myristoylation sites, whereas AhDGAT2b contained only three. Moreover, the three-dimensional structure of AhDGAT2b contained three beta strands (amino acid positions 22–23, 211–214, and 265–267) that were absent in AhDGAT2a (Figure 3). We speculated that these motif and structural differences could lead to differences in function. Hence, we constructed AhDGAT2a and AhDGAT2b plasmids to enable us to investigate their individual functions in *E. coli*.

**Figure 3:** Predicted two and three-dimensional structures of AhDGAT2a and AhDGAT2b. Structures were predicted using phyre2 (http://www.sbg.bio.ic.ac.uk/phyre2/html/page.cgi?id=index). (A, B) Predicted two-dimensional structures of AhDGAT2a and AhDGAT2b, respectively. (C, D) Predicted three-dimensional structures of AhDGAT2a and AhDGAT2b. The rainbow coloration indicates the progression from N (red) → C (indigo) terminus.

**Table 1:** Putative functional motifs in peanut AhDGAT2s predicted by PROSCAN.

Functional site	AhDGAT2a		AhDGAT2b	
	Position	Amino acid	Position	Amino acid
N-glycosylation	6–9	NVTA	6–9	NVTV
cAMP- and cGMP-dependent protein kinase phosphorylation	90–93	RKLS	90–93	RKLS
Protein kinase C phosphorylation	29–31	SSK	29–31	SSK
	118–120	SNR	118–120	SNR
	178–180	TKK	178–180	TKK
Casein kinase II phosphorylation	184–187	SLLD	184–187	SLLD
	298–301	TTEE	298–301	TTEE
	312–315	SLQD	312–315	SLQD
N-myristoylation	5–10	GNVTAA	–	–
	173–178	GLTPAT	173–178	GLTPAT
	198–203	GVQETF	198–203	GVQETF
	208–213	GTETAY	208–213	GTETAY
Amidation	88–91	FGRK	88–91	FGRK

### AhDGAT2a and AhDGAT2b fusion proteins are located in both soluble and insoluble fractions of *E. coli* cells

The AhDGAT2a and AhDGAT2b fragments were inserted into pGEX-4T-1 expression vector, transformed into *E. coli*, and the recombinant AhDGAT2–GST proteins, containing a GST-tag at the N-terminus, were induced with IPTG at 25°C or 37°C. Recombinant AhDGAT2 expression at 25°C was somewhat lower than that at 37°C (data not shown), so we selected 37°C as the optimal induction temperature. Cells induced at 37°C were collected after 0, 2, 4, and 6 h and the recombinant proteins extracted for SDS–PAGE analysis (Figure 4). Recombinant AhDGAT2 expression increased over time and was highest at 6 h, so this time point was used for subsequent experiments. No obvious differences were detected between the AhDGAT2a and AhDGAT2b expression levels.

**Figure 4:** SDS–PAGE analysis of the time course for expression of AhDGAT2a and AhDGAT2b recombinant fusion proteins in *E. coli* cell extracts. Recombinant proteins transformed into *E. coli* were induced with IPTG and their expression levels evaluated after 0, 2, 4, and 6 h. Molecular weight standards are shown on the left. The relative mobilities of GST (26.97 kDa), AhDGAT2a–GST (64.5 kDa), and AhDGAT2b–GST fusion proteins (64.5 kDa) are indicated on the right.

Following IPTG induction of the AhDGAT2 proteins, their production was scaled up to facilitate purification from the cytoplasmic fraction and inclusion bodies. Fusion proteins were purified and loaded onto SDS–PAGE for analysis (Figure 5). The fusion proteins were present in both the soluble (cytoplasm) and insoluble (inclusion bodies) fractions, with the largest quantities present in the inclusion bodies. The expression patterns of AhDGAT2a and AhDGAT2b did not differ noticeably.

**Figure 5:** Expression of AhDGAT2–GST fusion proteins after induction with 1 mM IPTG at 37°C for 6 h. M: Protein molecular weight marker. (A) Lanes 1, 3: AhDGAT2a–GST and AhDGAT2b–GST extracted from the cytoplasmic fraction; Lanes 2, 4: AhDGAT2a–GST and AhDGAT2b–GST extracted from inclusion bodies. (B) Western blot analysis of the AhDGAT2–GST fusion proteins using anti-GST tag monoclonal antibody. Lane 1: Wild-type *E. coli* Rosetta (DE3) strain; Lane 2, GST expression from the empty-vector transformed strain; Lanes 3, 5: AhDGAT2a–GST and AhDGAT2b–GST from the cytoplasmic fraction; Lanes 4, 6: AhDGAT2a–GST and AhDGAT2b–GST from inclusion bodies.

### Overexpression of AhDGAT2s affects the growth rate and morphology of transformed *E. coli*

Expression of GST or AhDGAT2–GSTs depressed the growth rate of the *E. coli* Rosetta (DE3) strain relative to the WT strain (Figure 6). This result was not unexpected, because carrying a foreign vector or expressing a foreign gene is likely to retard bacterial growth rates. After IPTG was added to the medium, the reduction in growth rate became more obvious. After 5 h in culture, the growth rate of the WT *E. coli* reached a plateau, whereas the growth rates of the three transformed lines increased for up to 7 h and showed no apparent differences among one another.

**Figure 6:** Growth curves of the wild type and transformed *E. coli* strains in liquid culture. The optical density (OD_600_) of the bacterial cultures is shown on the y axis. Bacteria were incubated aerobically at 37°C with shaking at 170 rpm. Vertical bars represent the standard deviation of three replicates.

We also studied the morphology of the *E. coli* strains before and after IPTG induction. Overexpression of both AhDGAT2a–GST and AhDGAT2b–GST substantially affected the morphology of the transformed *E. coli* cell lines (Figure 7; Table 2). Before IPTG induction, the WT and transformed *E. coli* lines showed no obvious differences in size or shape (Figure 7A,C,E,G). Unlike the WT line, which was unaffected by IPTG (Figure 7A–B), the empty-vector transformed line formed long filamentous structures instead of normal short rods within 2 h of IPTG induction. The filament lengths increased over time, and after 6 h of IPTG induction, the cell volume had significantly increased by about 1.5 times that of the un-induced control (Figure 7D; Table 2, *P<*0.05). The same phenomenon was observed in *E. coli* cells harboring AhDGAT2a–GST or AhDGAT2b–GST. The AhDGAT2a–GST and AhDGAT2b–GST vector-transformed cells increased markedly in size after IPTG addition, by ∼2.4–2.5 times (*P*<0.01) (Table 2; Figure 7F,H). Differences between AhDGAT2a–GST and AhDGAT2b–GST vector-transformed cells were less obvious. Of note, the length but not the width of the transformed *E. coli* cells increased (Table 2).

**Figure 7:** Morphology of wild type and transformed *E. coli* before and 6 h after the addition of IPTG into the growth medium. Cells were sampled and Gram stained before induction (A, C, E, G) and 6 h after induction (B, D, F, H). (A, B) wild-type *E. coli* cells; (C, D) empty-vector transformed cells; (E, F) AhDGAT2a–GST vector transformed cells; (G, H) AhDGAT2b–GST vector transformed cells.

**Table 2:** Cell sizes (mean±SE) of the recombinant *Escherichia coli* strains.

		WT strain	Empty vector	AhDGAT2a–GST	AhDGAT2b–GST
Uninduced cells	width ( µm)	4.10±0.12	4.08±0.14	4.08±0.13	4.07±0.11
	length ( µm)	27.198±4.90	25.913±3.42	27.841±4.95	27.626±3.99
	volume ( µm^3^)	358.90±61.57	341.95±42.91	367.38±62.19	364.55±50.14
Induced cells (6 h)	width ( µm)	4.11±0.13	4.12±0.14	4.08±0.13	4.11±0.12
	length ( µm)	27.412±4.23	41.975±7.09 a	66.175±5.16 b	67.032±10.37 b
	volume ( µm^3^)	361.73±53.15	553.90±89.08 a	873.23±64.77 b	884.54±130.2 b

a: Significantly different from WT at the 0.05 level.

b: Significantly different from WT at the 0.01 level.

### AhDGAT2 overexpression significantly affected the FA content of *E. coli* cells

The FA content of the IPTG-induced WT and transformed strains and their corresponding controls were analyzed by gas chromatography. Twenty-two types of FA were detected in the WT and transgenic *E. coli* strains (Table S1), with five main types accounting for 82.10–88.68% of the total FA content. C16:0 was the most abundant FA, comprising 45.52–61.5% of the total FA content. The other common FAs were C18:3n3 (12.42–19.88% of the total FA abundance), C14:0 (8.83–10.14%), C18:2n6t (6.46–9.01%), and C12:0 (4.91–5.94%). The contents of the remaining 17 FAs were below (0–8.34%).

In most cases when cell strains were un-induced, the empty-vector transformed *E. coli* strain showed no significant differences in FA content compared with the WT (Figure 8). Remarkably, transformation with AhDGAT2a–GST and AhDGAT2b–GST significantly increased the total FA content of the strains by 15.2–19.0% compared with the WT (*P*<0.01; Figure 8A) and also significantly affected some individual FA levels. The quantities of C14:0, C16:0, C16:1, and C18:1n9c showed significant increases compared with either the WT or empty-vector transformed strains (Figure 8C,E,F,G; *P<*0.01 or 0.05). The quantities of C12:0, and C18:3n3 showed significant increases only under IPTG induction compared with either the WT or empty-vector transformed strains (Figure 8B, I; *P<*0.01 or 0.05). The levels of C15:0 decreased significantly relative to the WT in both uninduced (*P*<0.01) and induced (*P*<0.05) AhDGAT2a–GST and AhDAGT2b–GST strains (Figure 8D), while the levels of C21:0 decreased significantly in the uninduced strains (*P<*0.01) and increased significantly in the induced AhDGAT2a strain (*P*<0.05; Figure 8J). However, the C18:2n6t content remained unchanged, except for a decrease in the uninduced AhDGAT2a–GST strain (*P*<0.05; Figure 8H).

**Figure 8:** Fatty-acid content of wild-type *E. coli* strains and strains transformed with empty vector, AhDGAT2a–GST, and AhDAGT2b–GST. Open columns represent the values in un-induced strains and filled columns the values in IPTG-induced cultures after 6 h. Vertical bars represent the standard deviations of three replicates. a,c,e, significant at the 0.05 level; b,d,f, significant at the 0.01 level. a and b, compared with WT; c and d, compared with the empty-vector strain; e and f, compared with AhDGAT2a-GST vector strain. *P* values are given in Table S1.

The effect of IPTG induction on the FA content of the different *E. coli* lines was also examined (Figure 8). The quantities of the individual FAs differed dramatically between the induced cultures and the WT. The C12:0, C14:0, C18:3n3, and C21:0 FA contents increased significantly (Figure 8B,C,I,J). In the AhDGAT2a–GST transformants, the respective increases were 10.06%, 3.63%, 40.38%, and 311.54%, and in the AhDGAT2b–GST transformants, the increases were 6.74%, 6.37%, 52.77%, and 240.91%, respectively (Table S1). In contrast, the C16:0, C16:1, and C18:1n9c contents decreased substantially after IPTG induction (Figure 8E,F,G). In the AhDGAT2a–GST transformants, the decreases were 9.45%, 88.09%, and 16.67%, respectively, while the AhDGAT2b–GST transformants decreased by 5.34%, 89.08%, and 35.56%.

The transformants carrying AhDGAT2a and AhDGAT2b also differed in their contents of some FAs, indicating possible functional differences between the two genes. When uninduced, the levels of C12:0 (*P*<0.05), C18:2n6t (*P*<0.01), CLA-c9t11 (*P*<0.01) (Figure 8B,H,K), and C22:ln9 (*P*<0.05) (Figure 8L) were significantly higher in the AhDGAT2b strain than in the AhDGAT2a strain. When induced, the AhDGAT2b strain contained significantly more C18:3n3 and C15:0 (*P*<0.01) (Figure 8I,D) and significantly less C21:0 and C22:ln9 (*P*<0.05) (Figure 8J,L).

## Discussion

### Overexpression of AhDGAT2 increases the FA content of *E. coli* cells

Increasing energy costs and environmental concerns have compelled the production of sustainable renewable fuels and chemicals. In recent years, biofuels have received significant attention and investment [27]–[35]. Prokaryotic expression systems, particularly *E. coli* systems, remain an effective way of producing large quantities of a variety of fusion proteins. For example, Lu et al. introduced four distinct genetic changes into the *E. coli* genome to achieve a high level of FA production (2.5 g/L) [27]. Zhang et al. studied the effects of overexpression of acyl-ACP thioesterase genes from four different plant species using *E. coli* that lacked FA production, and found that the transformed *E. coli* strains synthesized approximately 0.2 g/L of free FAs [35]. Jeon et al. cloned and overexpressed five genes (acetyl-CoA carboxylase A, acetyl-CoA carboxylase B, acetyl-CoA carboxylase C, malonyl-CoA-[acyl-carrier-protein] transacylase, and acyl-ACP thioesterase) in *E. coli* MG1655 and found that the FA (C16) levels from the recombinant strains were 1.23–2.41 times higher than those from the wild type [34]. Furthermore, Liu et al. engineered an *E. coli* cell line that produced 4.5 g/L/day FAs [33]. In addition, when a soluble DGAT3 from peanut was introduced into *E. coli*, the transformants showed high levels of DGAT activity and formation of labeled TAG [5].

In this study, we overexpressed two types of AhDGAT2 in *E. coli* Rosetta (DE3) and showed that the FA content of the transformants was significantly higher than in the WT or empty-vector transformed strains (increases from 15.18–18.94%; Table S1). The 6 h induction time used in our experiment was shorter than in most previous reports (5–48 h) [27], [34], [35]. Some reports have stated that the FA content and composition of certain *E. coli* strains (e.g. ML103 (pXZCO16, pXZ18, and pXZJ18)) changes over time [35]. We do not know whether the FA content of the AhDGAT2-transformed *E. coli* strains would increase with longer induction times, but our study clearly demonstrated the potential of AhDGAT2 for efficient FA production in *E. coli.*

### Overexpression of AhDGAT2 in *E. coli* changed its morphology

Bacteria have evolved sophisticated systems to maintain their morphologies. However, in certain environments, rod-shaped bacteria can become more filamentous [36]. Numerous bacteria alter their shapes in response to the types and concentrations of internal and external compounds. For example, the *E. coli* DH5α strain forms long filamentous cells upon caffeine exposure [37], while over-production of penicillin-binding protein 2 causes morphological changes and lysis in *E. coli* [38]. Nutritional stress most frequently induces filamentation, which can increase the total surface area of a bacterium without increasing its width; hence its surface-to-volume ratio does not change [39].

In this study, the transformed *E. coli* strains changed their general morphology from short rods to filamentous structures (Figure 7), a change similar to bacteria encountering nutritional stress [39]. These changes occurred gradually over time (data not shown) and were not caused by IPTG addition alone, because IPTG induction over 6 h caused no such morphological changes in the WT strain (Figure 7A–B). Furthermore, when fresh medium with or without IPTG was added to the 6-h induced cultures, the cells neither increased nor decreased in length when IPTG was included in the fresh medium, but they gradually shortened over several hours when IPTG was absent from the fresh medium (data not shown), suggesting that nutritional stress did not cause the changes in morphology. Perhaps the rapid accumulation of over-expressed proteins or FAs altered the cell shape. To some extent, cell size was related to the size of exogenous proteins produced. For example, GST transformants that produced ∼27 kDa proteins had cell sizes about 1.5 times those of their uninduced counterparts (Table 2). In contrast, AhDGAT2a–GST and AhDGAT2b–GST transformants (expressing 64 kDa AhDGAT2–GST fusion proteins) increased their sizes by about 2.4–2.5 times that of their uninduced counterparts (Figure 7E–F, G–H). Apparently, the larger the size of the exogenous protein, the larger the transformed cell will become.

### IPTG induction and FA content in *E. coli*

Zhang et al. examined the effect of IPTG concentration on free FA accumulation and found that total free FA accumulation responded in a dosage-dependent way up to 500 µM of IPTG [35]. Below 500 µM, the cultures accumulated similar quantities of free FAs [35]; above this value, the percentages of the C14 and C16:1 straight chain FAs increased markedly, whereas the percentages of C16 and C18 fell dramatically [35]. In our study, IPTG affected FA accumulation in *E. coli*. The cellular content of the individual FAs differed dramatically between the un-induced and induced cultures (Figure 8). The C12:0, C14:0, C18:3n3, and C21:0 cell contents increased significantly, whereas the C16:0, C16:1, and C18:1n9c contents decreased significantly. Furthermore, the transformants with AhDGAT2a and AhDGAT2b showed significant differences in the production of some FAs, suggesting that these two isozymes have slightly different functions in peanut plants. We did not examine whether different IPTG concentrations affected cellular FA levels; however, our finding that IPTG induction altered FA content was consistent with that of Zhang et al. [35].

## Conclusions

In this study, we cloned and successfully expressed the peanut DGAT2 genes in *E. coli.* The integral membrane proteins accumulated in the cells at a high level after IPTG induction, and the levels of several FAs were significantly higher in transformed cells, offering the possibility that these high-energy molecules might someday be generated for energy. In addition, we established an efficient way to express an integral membrane protein in *E. coli* that future studies can follow. We also identified the function of the peanut DGAT2 enzyme in *E. coli.*

Furthermore, the identification of these genes will help spur the creation of transgenic peanut germplasms with high oil content or other special characteristics. The DGAT antibody will be important for identifying DGAT protein expression levels in transgenic plants. Finally, the differences in enzyme activity *in vitro* will assist in identifying important motif sites or single nucleotide polymorphisms that can be used in molecular marker-assisted breeding.

## Supporting Information

Figure S1 **Comparison of the nucleotide sequences of** ***AhDGAT2a*** **and** ***AhDGAT2b*** **.** The 14 nucleotide differences are shaded in gray. The red underlines show the initiation and termination codons.
(TIF)

Table S1 **Original data and data analysis.**
(XLS)
